# Effect of Exercise Intervention on Internet Addiction and Autonomic Nervous Function in College Students

This article has been retracted.

**DOI:** 10.1155/2022/5935353

**Published:** 2022-09-05

**Authors:** Wei Zhang, RuiLin Xu

**Affiliations:** Zhengzhou University, Institute of Physical Education (School Headquarters), Henan Zhengzhou 450000, China

## Abstract

**Objective:**

To investigate the effects of 12-week physical exercise (jogging, basketball, and outdoor training) on sleep quality, harmful mood, and heart rate variability (HRV) in college students with Internet addiction.

**Methods:**

46 college students with Internet addiction were chosen and then randomly assigned to the Internet addiction group (IA, *n* = 23) and the Internet addiction exercise group (IA+EX, *n* = 23). The subjects in the IA+EX group underwent physical exercise for 12 weeks (three times per week), and the IA group did not perform regular physical exercise during the experiment. Then, the degree of Internet addiction, depression, and sleep quality were evaluated by using Young's Internet Addiction Test (IAT) scale, Center for Epidemiologic Studies Depression (CES-D) scale, and Pittsburgh sleep quality index (PSQI); HRV were measured by using Polar Team 2 before and after physical exercise intervention.

**Results:**

(1) After the 12-week exercise, compared to preexercise intervention, the scores of IAT, CES-D, and PSQI significantly decreased (*t* = 12.183, 9.238, 5.660; *P* < 0.01) in the IA+EX group; compared with the IA group, the scores of IAT, CES-D, and PSQI significantly decreased (*t* = 2.449, 3.175, 4.487; *P* < 0.05, *P* <0.01) in IA+EX group college students with Internet addiction. (2) After the 12-week exercise, compared to preexercise intervention, LFn and the ratio of LF/HF significantly decreased (*t* = 5.650, 3.493; *P* < 0.01) and HFn significantly increased (*t* = −2.491, *P* < 0.05) in the IA+EX group; there were no significant differences in the above indexes before and after the experiment in the IA group (*P* > 0.05). Compared with the IA group, HFn significantly increased (*t* = 3.616, *P* < 0.01) and the ratio of LF/HF significantly decreased (*t* = 2.099, *P* < 0.01) in IA+EX group college students with Internet addiction; there was no significant difference in LFn between the two groups.

**Conclusion:**

Long-term physical exercise could significantly reduce the degree of Internet addiction and depression, improve sleep quality, and balance sympathetic parasympathetic function of college students with Internet addiction, indicating that exercise-based intervention might be an effective way to alleviate or even eliminate Internet addiction.

## 1. Introduction

According to the 2019 report of the China Internet Network Information Center, the number of Internet users in China reached 854 million, most of which are teenagers and young adults [1]. Although the Internet has brought great convenience to our lives, poor network usage can lead to impaired mental health, academic failure, decline in job performance, and especially Internet addiction. Internet addiction is a type of behavioral addiction, which refers to the uncontrolled online impulse under the influence of nonaddictive substances and manifests as a significant decline in social and psychological functions due to excessive use of the Internet [2]. Moreover, Internet addiction has been considered a serious mental disorder, which may lead to attention deficit, social phobia and impulsivity, depression, anxiety, and obsessive-compulsive disorder [3]. The investigation of Younes et al. [4] showed that Internet addiction could significantly affect the sleep quality, emotional disturbance, and self-esteem of college students, hindering their learning and affecting long-term career goals, which have produced extensive and harmful consequences for the whole society. Nowadays, these serious problems have attracted widespread attention in society and the research on the underlying mechanisms of Internet addiction and mood disorders is urgently needed. Studies have shown that Internet addiction is closely related to autonomic dysfunction. The heart rate variability (HRV) is an effective noninvasive measure to assess autonomic function by analyzing the frequency and time components of heart rate changes over time. Lin et al. [5] found that the HRV decreased in children with Internet addiction, which was manifested as a significant increase in low-frequency power (LF) and a significant decrease in high-frequency power (HF) and total power (TP) which was associated with sleep disturbances in children with Internet addiction. And Kim et al. [6] found that adolescent autonomic dysfunction was related to depression caused by Internet addiction. In addition, Wang et al. [7] also found that the scores of the addiction scale for Internet addicts were positively correlated with LF and LF/HF ratio of HRV and negatively correlated with HF, which suggested that HRV can be used to assess whether adolescents are addicted to the Internet and is an important reference indicator of the severity of Internet addiction.

Meta-analysis shows that drug treatment (bupropion, methylphenidate, etc.), cognitive behavioral therapy, family group therapy, and active physical exercise have good effects on Internet addiction [8], among which exercise intervention is the low-cost and simple intervention method that has attracted much attention. Studies have shown an inverse relationship between physical activity levels and the severity of video game-related problems and Internet addiction [9]. And Cerrillo-Urbina et al. [10] found that physical exercise interventions can reduce inattention, hyperactivity, and impulsivity, as well as improve anxiety, executive function, and social skills in people with ADHD. In addition, Cao [11] found that yoga can improve the anxiety and depression of obese female college students by regulating the level of autonomic nervous function and promoting the physical and mental development of college students. And physical exercise can produce a series of pleasant feelings to the body, which can better eliminate the anxiety and depression of the body, make the body produce a great sense of happiness, and improve the mental health of the body. Based on the above literature, it can be seen that physical exercise intervention may have a positive effect on Internet addicts, but whether the effect of exercise on Internet addiction, bad mood, and sleep quality of college students with Internet addiction is related to the autonomic function needs to be confirmed by research. Therefore, the current study investigates the effect of a 12-week exercise intervention (jogging, basketball exercise, and outreach training) on sleep quality, negative emotions (anxiety and depression levels), and HRV in college students with Internet addiction, so as to provide a theoretical basis for exercise intervention on Internet addiction.

## 2. Objects and Methods

### 2.1. Research Objects

Based on G power calculation, 46 college students with Internet addiction were consulted in the psychological counseling room of Zhengzhou University and randomly divided into two groups, the Internet addiction group (IA; *n* = 23) and the Internet addiction exercise group (IA+EX; *n* = 23). There were 20 males and 12 females in the IA group, with an average age of 19.61 ± 1.19 years and the net age of 3.96 ± 1.07 years. There were 18 males and 14 females in the IA+EX group, with an average age of 19.39 ± 1.73 years and the net age of 4.04 ± 1.11 years. There was no statistical significance in the comparison of basic information such as age, gender, and Internet age among the two groups of college students by independent samples *t*-test (*P* > 0.05).

The inclusion criteria are as follows: ① those who have been diagnosed as Internet addicts by standardized clinical interview and Internet addiction test and ② no history of taking psychotropic drugs in the 1ast month. Exclusion criteria are as follows: ① those with a history of serious physical or psychological problems, including other addiction disorders, psychotic disorders, and major depressive disorders; ② those with serious physical illnesses; and ③ students who are using drug therapy and are receiving psychological therapy. Before the intervention, all subjects filled out the informed consent form and the research purpose, process, benefits, and possible inconveniences are explained in detail to the subjects, and it was approved by the ethics committee of the university.

### 2.2. Methods

#### 2.2.1. Exercise Intervention Program

From September to November 2020, exercise intervention was implemented in Zhengzhou University for 12 weeks (3 times/week, 60 min/time). Each exercise includes 10 minutes of warmup, 10 minutes of relaxation exercises (jogging and stretching), and 40 minutes of aerobic exercise, including jogging, basketball exercise, and outreach training (exercise intensity: 60%-65% HRmax). In order to ensure the safety during exercise, the Polar Sports tester monitors the exercise intensity of the subjects. The control group was sedentary at the same time, and the members of the experimental group recorded their feelings of daily exercise.

#### 2.2.2. Adolescent Internet Addiction Scale

Before and after the exercise intervention, all subjects were used to assess the severity of compulsive Internet use by the Young's Internet Addiction Test (IAT) which is widely used in international studies, and its validity and reliability have been proved in previous studies. The scale included 5 components and 20 items and is scored on a 5-point Likert scale (1 is hardly ever, 2 is occasionally, 3 is sometimes, 4 is often, and 5 is always); the total score is 100 points, 40-60 is mild Internet addiction, 60-80 is moderate Internet addiction, and 80-100 is severe Internet addiction. This scale has high reliability and validity; Cronbach's alpha coefficient is 0.90 [12].

#### 2.2.3. CES-D Self-Rating Depression Scale

The CES-D scale is used to evaluate depressive symptoms in the general population and to screen people at high risk for depression. The scale has been tested in Chinese adolescents and achieved good reliability and validity. The scale contains a total of 20 items and is used to measure the frequency of depressive symptoms in the past week. The scale uses a 4-point scoring system (0 is hardly ever, 1 is sometimes, 2 is often, and 3 is most of the time), and the overall score ranges from 0 to 60 points, with higher scores for depression the higher the degree. A score of 0-15 indicates no depression, a score of 16-20 indicates mild depression, a score of 21-30 indicates moderate depression, and a score greater than 30 indicates severe depression. Cronbach's alpha coefficient of this scale is 0.86 [13].

#### 2.2.4. Pittsburgh Sleep Quality Index (PSQI)

Before and after the exercise intervention, the sleep status of the subjects within one month was assessed using a standard and valid questionnaire of the PSQI scale. The scale consists of 19 items, of which 18 items generated seven components (subjective sleep quality, sleep latency, sleep duration, habitual sleep efficiency, sleep disturbances, use of sleeping medication, and daytime dysfunctions), each of which is scored on a 0-3 scale (0 means very good, 1 means good, 2 means bad, and 3 indicates very poor), and the total score is 0-21 points. A total score of <5 indicates satisfactory sleep quality, and ≥5 indicates poor sleep quality. Cronbach's alpha coefficient is 0.74 [14].

#### 2.2.5. HRV Measurement

The HRV of subjects was measured using a Polar Team 2 team before and after exercise intervention. In order to avoid the influence of circadian rhythm on autonomic function, HRV measurement was scheduled at 8:00-10:00 am, the test environment humidity was 55-65%, and the temperature was 25 ± 1°C. Before the test, the experimenter should wear a chest strap, lie down, and rest for 10 minutes. The Polar 2 software for data collection was opened and gathered for 10 minutes when the subjects breathe calmly. *Test indicators include* low-frequency power (low frequency (LF), 0.04-0.15 Hz), high-frequency power (high frequency (HF), 0.15-0.4 Hz), and low-frequency/high-frequency (LF/HF) ratio.

### 2.3. Statistical Analysis

All experimental data are represented by $\bar{x}\pm s$, and the data was analyzed using SPSS 21.0 statistical software package. Normal distribution was analyzed using the Shapiro-Wilk test; since LF and HF do not obey normal distribution, statistical analysis is performed after logarithmic transformation (Ln). Paired *t*-test was used to compare the experimental data before and after exercise intervention within the group (groups IA and IA+EX). Independent samples *t*-test was used to analyze the differences between groups in IAT, CES-D, and PSQI scores and HRV indexes before and after exercise intervention, and *P* < 0.05 indicated that the difference was statistically significant.

## 3. Results

### 3.1. The Effect of Exercise Intervention on Internet Addiction and Depression in College Students with Internet Addiction

As shown in Table 1, compared with preexercise, the scores of IAT and CES-D of college students in the IA+EX group significantly decreased (*t* values were 12.183 and 9.238; *P* < 0.01), and the decrease was 10.35% and 8.74%, respectively; there was no significant difference in the above indicators in the IA group before and after the experiment (all *P* > 0.05). Before the exercise intervention, there was no significant difference in the scores of Internet addiction and depression between the college students in the IA+EX group and the IA group (*t* values were -0.502 and -0.434, *P* > 0.05); after the exercise intervention for 12 weeks, compared with the IA group, the scores of Internet addiction and depression level of college students in the IA+EX group significantly decreased (*t* values were 2.449 and 3.175; *P* < 0.05 and *P* < 0.01).

### 3.2. The Effect of Exercise Intervention on the Sleep Quality of College Students with Internet Addiction

As shown in Table 2, after 12 weeks of exercise intervention, compared with preexercise, the scores of subjective sleep quality, sleep latency, sleep disturbance, and daytime dysfunction in college students with Internet addiction significantly decreased (*t* values were 2.577, 2.313, 2.152, 2.472, and 5.660; *P* < 0.05 and *P* < 0.01); there was no significant change in sleep persistence, habitual sleep efficiency, and hypnotic drug dependence before and after intervention in the IA+EX group (*t* values were 1.367, 1.447, and 1.000; *P* > 0.05); all the above indexes in the IA group had no significant changes before and after the experiment (*P* > 0.05). Before exercise intervention, there were no significant differences in the scores of 7 components of sleep quality and PSQI between the IA group and the IA+EX group (*P* > 0.05). Except the scores of subjective sleep quality, sleep latency, sleep disturbance, daytime dysfunction, and PQSI significantly decreased (*t* values were 2.275, 2.053, 2.065, 2.655, and 4.487; *P* < 0.05 and *P* < 0.01). There was no significant difference in the scores of habitual sleep efficiency and hypnotic drug dependence when compared with the IA group (*t* values were 1.164, 1.026, and -0.321; *P* > 0.05).

### 3.3. Effect of Exercise Intervention on HRV of College Students with Internet Addiction

As shown in Table 3, after 12 weeks of exercise intervention, compared with preexercise, the LFn and LF/HF of college students with Internet addiction in the IA+EX group significantly decreased (*t* values were 5.650 and 3.493; both *P* < 0.01); the decrease was 3.87% and 34.45%, respectively; HFn significantly increased by 2.25% (*t* = −2.491, *P* < 0.05); there was no significant difference in all the above indexes before and after the experiment in group IA (*P* > 0.05). There were no significant differences in LFn, HFn, and LF/HF between the IA group and the IA+EX group before exercise intervention (*t* values were -0.216, 0.435, and 0.471; *P* > 0.05); after 12 weeks of exercise intervention, compared with the IA group, the HFn of IA+EX college students with Internet addiction increased significantly (*t* = 3.616, *P* < 0.01), and the LF/HF ratio decreased significantly (*t* = 2.099, *P* < 0.05). There was no significant difference in LFn between the two groups (*t* = 2.099, *P* < 0.05; *t* = −0.792, *P* > 0.05).

## 4. Discussion

### 4.1. The Effect of Exercise Intervention on Internet Addiction, Depression, and Sleep Quality of College Students with Internet Addiction

The Internet has become a key resource in society and everyday life, and Internet addiction is another worldwide public health problem. Internet addiction has also been considered as a psychological escape mechanism to avoid real-world problems and has been proven to be associated with both mental and physical symptoms. Examples are the higher risk of Internet addition, inferior mental health outcomes, suicidal ideation, depression, and anxiety [15]. Meta-analysis shows that the global prevalence of Internet addiction is 1.6%-18% [16], while the prevalence of Internet addiction among Chinese college students is 11.3% [17]. The negative impact of Internet addiction on physical and mental health has been a major public concern. It is reported that Internet addiction is significantly associated with mood disorders, poor sleep quality, low self-esteem, impulsivity, suicide, low levels of physical activity, and health problems (migraines, back pain, and obesity), and the prevalence of poor sleep quality, depression, and anxiety symptoms is high among college students worldwide [18]. In addition, college students with sleep problems are more likely to have symptoms of depression. In recent years, physical exercise as an alternative or adjunctive treatment for Internet addiction has been extensively studied. Meta-analysis showed that exercise intervention significantly improved various dimensions of the Internet addiction scale and psychopathological symptoms, especially the improvement of Internet addiction symptoms [19]. In addition, Internet addiction is related to decreasing physical activity by the Internet addiction scale. Compared with physical inactive peers, physical active young people tend to get more satisfaction from sleep and are less likely to develop Internet addiction [20]. And Kocak [21] found that regular exercise (12 weeks, 3-5 times/week, at least 45 min/time) can reduce college students' Internet addiction and Internet time and help to prevent the psychosocial, physical, and psychological negative effects induced by Internet addiction, which suggested that regular physical exercise can reduce and prevent college students' Internet addiction. The research of Zheng et al. [22] suggested that exercise intervention has a positive effect on the treatment of smartphone addiction and should be regarded as an alternative nondrug method for the treatment of smartphone addiction patients. In addition, Wang et al. [23] thought that at least 12 weeks of physical exercise can lead to the adaptation of key brain structures involved in reward and inhibitory control and improve Internet addiction symptoms. And physical exercise especially moderate-intensity comprehensive sports intervention (basketball, badminton, sports games, etc.) has been confirmed to be better improvement in the prevention and treatment of Internet addiction [24]. Therefore, the current study implemented a 12-week exercise intervention (including jogging, basketball, and expansion sports) for the Internet addicts. The results showed that compared with the IA group, the scores of Internet addiction and depression levels of college students in the IA+EX group significantly decreased, and the sleep quality significantly improved, indicating that exercise intervention may be an effective way to alleviate or even eliminate Internet addiction. However, Gao et al. [25] found that an 8-week exercise intervention has a good effect on the mental health correction in mild Internet addicts, but the treatment effect is not ideal for moderate and severe patients. The current study mainly recruited mild and moderate Internet addicts, and further research needs to conduct exercise intervention studies on Internet addicts with different degrees.

### 4.2. The Effect of Exercise Intervention on HRV of College Students with Internet Addiction

The substantial association between both Internet addiction and depression and sleep quality and social support may shed insights to our understanding about the mechanism. HRV is directly controlled by the central nervous system and the autonomic nervous system, and it is one of the important indicators of the human body's adaptation process, but there are few reports on the effects of Internet addiction on autonomic nervous function. The results of this study found that college students with Internet addiction had higher sympathetic nerve activity and lower parasympathetic nerve activity and overall autonomic nerve activity, which suggested that long-term, excessive use of the Internet is at risk of reducing HRV levels. Studies have shown that HRV is an effective tool for measuring and regulating emotional responses, and the reduction in HRV indicates autonomic dysregulation and lack of flexibility in response to stimuli, which can lead to physical and psychological disorders (emotional dysregulation and decreasing social engagement) [26]. In the treatment of patients with anxiety and depression, Kircanski et al. [27] found that patients with high HRV have a better prognosis, while those with low HRV have a poorer prognosis, indicating that HRV has broad application prospects in evaluating the prevention of psychosomatic and mental dysfunction/the therapeutic effect of intervention. Therefore, it can be considered that the depression level of college students with Internet addiction in this study may be related to the reduction of HRV. However, the mechanism of the reduction of HRV in the college students with Internet addiction is still unclear. Kim et al. [6] thought that Internet addiction can change the sleep-wake schedule, so excessive use of the Internet will deprive sleep time of people, which results in poor sleep quality and exerts adverse effects on autonomic nervous system function. And Lin et al. [28] found that Internet addiction is associated with higher sympathetic nerve activity and lower parasympathetic nerve activity, and lack of sleep (less sleep time and poor sleep quality) can activate the stress system and increase the catecholamine, norepinephrine, and epinephrine levels, thereby increasing sympathetic nerve activity, which suggests that the autonomic dysregulation associated with Internet addiction may be partly due to poor sleep quality. This study is a cross-sectional study and cannot confirm a causal relationship between Internet addiction, sleep quality, and the autonomic nervous system. In conclusion, the effect of Internet addiction on the autonomic nervous system function may be a comprehensive effect of psychological, physiological, and behavioral changes accompanying Internet overuse, and the mechanism of autonomic dysregulation associated with Internet addiction needs to be further elucidated.

Long-term physical activity has been shown to induce resting bradycardia with reducing sympathetic and/or elevated parasympathetic activity [29]. In addition, there is growing evidence that regular physical activity may enhance physical and mental health and relieve stress states by optimizing HRV and improve well-being [30]. Toni et al. [31] found that the combination of long-term physical exercise and the antidepressant sertraline could significantly increase HRV in elderly patients with depression and had an antidepressant effect by regulating the cardiac autonomic function. And Tseng et al. [32] found that 12 weeks of moderate-intensity exercise training had a beneficial effect on sleep quality and cardiac autonomic function; middle-aged and elderly people with poor sleep quality should be encouraged to perform moderate-intensity aerobic exercise to improve their cardiac autonomic function. In addition, Zhang et al. [33] found that 24-week aerobic exercise can reduce drug addiction of drug addicts by regulating the autonomic nervous function of compulsory drug addicts. However, there are few related reports on the effect of exercise on the HRV of college students with Internet addiction. The results of this study found that compared with the IA group, after 12 weeks of exercise intervention, the HFn increased significantly and the LF/HF ratio decreased significantly of college students with Internet addiction in IA+EX, indicating that long-term physical exercise may improve the excitability of the vagus nerve and promote sympathetic-parasympathetic balance, which can improve the cardiac autonomic function of college students with Internet addiction to a certain extent. In addition, it was previously reported that low HRV was significantly associated with self-regulation ability and craving for Internet use [34]. Therefore, the improvement of long-term physical exercise on Internet addiction in college students with Internet addiction is related to the increase of HRV and the balance of sympathetic-parasympathetic nerve function.

## 5. Summary

The increase of HRV can enhance the emotion regulation ability and improve the level of depression and sleep quality of the college students with Internet addiction, and the specific mechanism needs to be further studied.

## Figures and Tables

**Table 1:** Results of IAT and CES-D scores in college students with Internet addiction before and after the exercise interventions $\left(\bar{x}\pm s\right)$.

Group	Before and after	*n*	Value	CES-D	IAT
IA group	Before	23		26.78 ± 5.63	66.83 ± 6.26
	After	23		27.83 ± 5.72	67.91 ± 7.12
			*t* value	−1.850	−1.150
			*P* value	0.078	0.262
IA+EX group	Before	23		26.96 ± 4.80	68.09 ± 10.29
	After	23		24.17 ± 5.47^∗∗^^#^	62.14 ± 8.81^∗∗^^#^
			*t* value	9.238	12.183
			*P* value	0.000	0.000

Note: ^∗^*P* < 0.05 and ^∗∗^*P* < 0.01, significant difference before vs. after program; ^#^*P* < 0.05 and ^##^*P* < 0.01, the IA group vs. the IA+EX group.

**Table 2:** Results of PSQI scores in college students with Internet addiction before and after the exercise interventions $\left(\bar{x}\pm s\right)$.

Sleep quality (score)	Group	*n*	Before	After	*t* value	*P* value
Subjective sleep quality	IA	23	1.26 ± 0.45	1.30 ± 0.55	-0.569	0.575
	IA+EX	23	1.30 ± 0.70	0.96 ± 0.47^∗^^#^	2.577	0.017
Sleep latency	IA	23	1.17 ± 0.72	1.22 ± 0.67	-1.000	0.328
	IA+EX	23	1.13 ± 0.63	0.86 ± 0.46^∗^^#^	2.313	0.030
Sleep persistence	IA	23	0.91 ± 0.59	1.00 ± 0.60	-1.447	0.162
	IA+EX	23	0.96 ± 0.47	0.83 ± 0.39	1.367	0.816
Habitual sleep efficiency	IA	23	0.35 ± 0.48	0.30 ± 0.47	1.000	0.328
	IA+EX	23	0.30 ± 0.47	0.22 ± 0.42	1.447	0.162
Sleep disturbance	IA	23	1.22 ± 0.67	1.35 ± 0.71	-1.817	0.083
	IA+EX	23	1.13 ± 0.63	0.96 ± 0.56^∗^^#^	2.152	0.043
Hypnotic drug dependence	IA	23	0.22 ± 0.42	0.26 ± 0.45	-0.569	0.575
	IA+EX	23	0.35 ± 0.49	0.30 ± 0.47	1.000	0.328
Daytime dysfunction	IA	23	1.39 ± 0.58	1.52 ± 0.59	-1.817	0.083
	IA+EX	23	1.30 ± 0.56	1.09 ± 0.51^∗^^#^	2.472	0.022
PSQI	IA	23	6.52 ± 1.41	6.82 ± 1.44	-2.077	0.050
	IA+EX	23	6.47 ± 1.23	5.17 ± 1.03^∗∗^^##^	5.660	0.000

**Table 3:** Results of HRV parameters in college students with Internet addiction before and after the exercise interventions $\left(\bar{x}\pm s\right)$.

HRV	Group	Before	After	*t* value	*P* value
LFn	IA	3.91 ± 0.17	3.93 ± 0.15	-1.849	0.060
	IA+EX	3.88 ± 0.18	3.73 ± 0.23^∗∗^	5.650	0.000
HFn	IA	3.55 ± 0.31	3.59 ± 0.28	-2.019	0.056
	IA+EX	3.57 ± 0.29	3.64 ± 0.30^∗^^##^	-2.491	0.021
LF/HF	IA	2.59 ± 1.58	2.62 ± 1.50	-0.208	0.837
	IA+EX	2.38 ± 1.42	1.56 ± 1.70^∗∗^^#^	3.493	0.002

## Data Availability

The experimental data used to support the findings of this study are available from the corresponding author upon request.
